RETRACTED

# Data Mining Algorithm for Physical Health Monitoring of Young Students Based on Big Data

**DOI:** 10.1155/2021/9962906

**Published:** 2021-05-11

**Authors:** Jiangang Sun, Xiaoran Jiang, Guoliang Yuan, Zhenhuai Chen

**Affiliations:** ^1^School of Physical Education, West Anhui University, Lu'an 237012, Anhui, China; ^2^School of Physical Education, Hengshui University, Hengshui 053000, Hebei, China; ^3^Faculty of Physical Education, China West Normal University, Nanchong 637000, Sichuan, China

## Abstract

With the continuous improvement of living standards, the level of physical development of adolescents has improved significantly. The physical functions and healthy development of adolescents are relatively slow and even appear to decline. This paper proposes a novel data mining algorithm based on big data for monitoring of adolescent student's physical health to overcome this problem and enhance young people's physical fitness and mental health. Since big data technology has positive practical significance in promoting young people's healthy development and promoting individual health rights, this article will implement commonly used data mining algorithms and Hadoop/Spark big data processing. The algorithm on different platforms verified that the big data platform has good computing performance for the data mining algorithm by comparing the running time. The current work will prove to be a complete physical health data management system and effectively save, process, and analyze adolescents' physical test data.

## 1. Introduction

In recent years, due to the rapid economic development, people spend more and more time at work and have less time for physical exercise and physical activity. All over the world, significant changes have taken place in the lifestyles of youths. This amount has been significantly reduced compared with before, and the busy schoolwork of adolescents has also led to a significant reduction in the time of their physical exercise [1]. In response to the current decline in young people and children's physical fitness, we are very concerned about adolescents' healthy development. We have adopted different scales and ranges of tests on students' physical fitness to understand and monitor the physical condition and urge improving the physical level. However, to make good use of such data is a problem, as well as how to use reasonable research methods to extend the research on deep-level logical relationships, analyze and summarize the data scientifically, and manage and reprocess the test data accordingly [2].

Moreover, utilization has always been a problem that society has not effectively solved, especially the accumulation of many young people's physical test data every year. Still, it has not been properly and effectively used [3]. On the one hand, it has caused a waste of data resources, and, on the other hand, it cannot be effectively utilized. Digging out the problems that the data can reflect, it is impossible to formulate a targeted intervention plan based on the corresponding data analysis results. Therefore, in the current environment of big data and deep learning [4], we should use data analysis systems to analyze and process data appropriately. The preservation, processing, and analysis of youth physical examination data have always been an essential part of its physical examination. The physical test score for young students still adopts a purely manual method; that is, after the physical test is completed [5], the score data is input or exported and saved as an Excel file.

RETRACTED

Some areas with more developed economies are more advanced, using instrument testing and wireless data transmission to connect with the education management department's system seamlessly. However, the data collected by the physical test must be currently only used for storage management [6]. Certain additions, deletions, and changes are made to the data, but it lacks effective use. The physical test data cannot provide real-time queries. The individual students and the school can also check the physical test data results, deeper understanding, and intuitive feeling. More importantly, the statistical analysis functions that can be achieved by the existing physical fitness test data management system are minimal [7].

This work will use commonly used data mining algorithms [8, 9] and Hadoop/Spark, a big data processing platform, to study and implement Hadoop/Spark-based structural health monitoring [10, 11]. By mining historical monitoring data and real-time monitoring data, a comprehensive analysis of young students' physical fitness is carried out. Comparing the algorithm's running time on different platforms shows that the big data platform has good computing performance for the data mining algorithm. This research aims to establish a complete physical health data management system and effectively save, process, and analyze adolescents' physical test data through the system. After the analysis, on the one hand, it can provide students and the school with intuitive analysis results. On the other hand, it can be accurate and reflect students' specific problems in physical health [12] to formulate specific measures to promote young people's physical fitness. The following are the main contributions of this paper:

1. Based on the Hadoop/Spark big data processing framework, this paper studies the data mining algorithm for adolescent students' physical health monitoring and uses data mining technology to analyze and mine adolescent students' physical health monitoring data
2. The Hadoop/Spark-based adolescent student physical health monitoring data mining algorithm can dig out practical information and knowledge from the adolescent student's physique data and real-time monitoring data, which has practical significance for research
3. We conducted simulation experiments, and the experimental results show that the algorithm in this paper effectively predicts young students' physical health

RETRACTED

## 2. Related Research

In this section, we will discuss the existing work in detail.

### 2.1. Youth Health-Related Research

According to the definition of health by the World Health Organization (WHO), individual health includes explicitly four aspects: physical health, mental health [13, 14], social interaction [15], and oral health [16]. At present, research on adolescent health issues is mainly carried out from the aspects of physical health and mental health. Research on adolescent health risk behaviors has gradually received researchers' attention with the deepening and expansion of study at home and abroad. Based on the research hotspots of adolescent health problems, this research divides the research of adolescent health problems into mental health research, physical health research, and health risk behavior research and comprehensively grasps adolescents' current health development status. Globally, the health risk behaviors of adolescents are very prominent. Early pregnancy and childbirth are endangering adolescents' health risks.

Similarly, reproductive health, interpersonal violence, and sexual violence bring about physical and psychological harm to adolescents. Besides, at least 1 in every ten young adolescents has smoking behavior; likewise, alcoholism weakens adolescents. Due to differences in socioeconomic [17] and cultural backgrounds, adolescents' health risk behaviors faced by different countries are different. However, these health risk behaviors are gradually endangering the foundation of adolescents' health.

For adolescents, the formation of their health literacy is more specific than that of adults. Parents and teachers are the primary source of health information and play a leading role in developing adolescents' health literacy, while health experts can only rank third. However, survey data from the National Bureau of Statistics of the United States found that parents' health knowledge and health abilities themselves are low, about 36%, and it is difficult to guide children and adolescents in healthy activities. The same data is less than 20% in China. The study found that the factors affecting adolescents' health literacy can be roughly classified into four categories: the influence of individual attributes, education system [18], health system, and family system [19].

RETRACTED

#### 2.1.1. Big Data

Big data refers to massive amounts of data with potential mining value. In the current information age, the widespread use of the Internet, the Internet of Things, cloud computing, and other emerging IT technologies have enabled various data sources to overgrow. At the same time, the structure and types of data have become more and more complex. With big data development, enterprises will upgrade and transform to the American Association for the Advancement of Science (AAAS) model [20], thereby changing IT and other industries' ecology. In this context, global giants in the IT industry (such as IBM, Google, Microsoft, and Oracle) have gradually launched technological development plans for the era of big data. The Big Data Research and Development Initiative, announced by the United States in March 2012, is a strategic plan to promote the United States' continuous leadership in the high-tech field and protect national security and promote social and economic development. At the same time, six federal government agencies, including the U.S. Department of Energy, have also taken action, jointly launching a big data research and development initiative, which aims to study new big data infrastructure and methods and improve the ability to use big data for scientific discovery. These technologies are used to accelerate the development of science and engineering, strengthen national security, completely change education and learning models, and vigorously cultivate new talents who develop and use big data technologies. In January 2013, the British government announced a £189 million big data plan. The plan aims to promote new opportunities for companies and research institutions to use big data and support further big data in medicine, industry, agriculture, and scientific research. Development of the Japanese government announced its national big data strategy, that is, Integrated Strategy for ICT in 2020” and “Becoming the World's Most Advanced IT Country” in 2012 and 2013, respectively. It plans to formulate big data as the core during 2013–2020, a new national IT strategy. Western countries represented by the United States are moving towards the modernization of their national power by researching and applying big data under their national agenda. The development of domestic significant data research is slower than that abroad. In December 2011, China released the “Twelfth Five-Year Plan” for the Internet of Things and began to develop critical technologies related to big data vigorously.

RETRACTED

Based on the research status and development trend of big data at home and abroad, it can be seen that big data has received extensive attention in various fields at home and abroad and has begun to flourish. Ahmad Jan et al. [21] discussed the application of big data technology in online structural health monitoring, using Spark instead of MapReduce technology, parallelized analysis, and calculation of infrared thermal imaging data of the structure, and realized damage diagnosis of the structure. According to the needs of structural health monitoring and the characteristics of monitoring data, Zhongdong Duan et al. [22] proposed a data mining framework for structural health monitoring, including task definition, data warehouse construction, data preprocessing, data mining, and program evaluation. Sung-Yan Park et al. analyzed the rate of physical activity participation in Korean adolescents by drawing significant implications based on terms and clusters through big data analysis [23]. These studies have explored the application of big data in structural health monitoring and have excellent application prospects. Lili Pan [24] developed a data mining tool for monitoring big data of physical exercises and sports. For this purpose, statistics and deep learning [25] were employed to collect and analyze competitive sports information.

## 3. Methodology

The details about methodology are provided below.

### 3.1. Adolescent Student Health Theory

The Adolescent Student Health Theory is divided into three parts. These parts are discussed in detail below.

#### 3.1.1. Subjective Evaluation of Individual Health

Health self-assessment has always been regarded as a primary way to grasp various groups of people's health status. It is widely used in existing citizen health surveys in China. There are five options in the self-assessment section of adolescent health: excellent health, reasonable, fair, chronic disease, and severe disease. The sample data shows that 332 people think that their health is excellent, accounting for 38.5% of the total number of samples, and 401 people think that their health is good, accounting for 46.5% of the total number of instances; in other words, more than 80% of teenagers believe that they are in good health. Besides, 12.5% of the research subjects rated their health as fair, and only 2.5% of the research subjects reported that they had chronic or severe diseases in the health self-evaluation, as shown in Table 1. On the whole, the self-evaluation of the health of the adolescents in the sample is very good.

#### 3.1.2. Physical Health

As an essential indicator of the adolescent health survey, physical health can most intuitively reflect adolescents' health status. The research design is based on the theoretical category of general health, starting from the myopia rate, sleep time, sports time, eating three meals, and so on, and, combined with adolescents' healthy living habits, a specific analysis of the adolescents' physical health is made. Among them, the sleep time is 7–8 hours a day as the health standard, the physical exercise time is half an hour to an hour of moderate-intensity exercise as the health standard, there is no partial eclipse, three meals are eaten on time as the diet health standard, and adolescents are investigated. The questionnaire includes five options, 1–5 points are never, occasionally, often, and always. Data analysis found that the average scores of the adolescents' sleep duration, physical exercise, and eating habits in the sample data were 3.16, 3.09, and 3.71, respectively, slightly higher than “sometimes,” but they did not meet the “frequent” health standards. The physical health and healthy living habits of adolescents need to be further improved, as shown in Table 2. For a more intuitive comparison, after further frequency analysis, it is found that 54.6% of teenagers sleep less than 7 to 8 hours per day, and more than 62.2% of teenagers spend less than half an hour per day in sports activities. 38% of young people have not developed good healthy eating habits.

RETRACTED

#### 3.1.3. Health Risk Behavior

In the existing research on the healthy development of adolescents, in addition to showing the status quo of the healthy development of adolescents from the dimensions of adolescents' physical health, mental health, and social interaction, foreign frontiers also attach great importance to the performance of adolescents' health risk behaviors. Adolescents' health-risk behaviors are opposite to health-promoting behaviors. According to Professor Ji's [26] research results, adolescents' health-risk behaviors can be divided into seven categories: accidental injury, intentional injury, substance addictive behavior, mental, addictive behavior, and unprotected sexual behavior. On the one hand, specific substance addiction behaviors include drug abuse, smoking, and drinking, and mental addiction behaviors include gambling, pornography addiction, and Internet addiction.

### 3.2. Principal Component Analysis-Based Abnormal Identification of Adolescent Students' Physical Health Monitoring

#### 3.2.1. Feature Extraction Based on the AR Model

In this section, we will discuss the feature extraction using AR model. The following equation can express the p-order autoregressive (AR) model:

(1) $$\begin{array}{c} x_{i}=\sum_{i=1}^{p}a_{i}x_{t-1}+\varepsilon_{t}, \end{array}$$

where *ε*_*t*_ is white noise, obeying *N*(0, *σ*^2^) distribution, *a*_i_ ∈ *Z*, *i*∈[1, p] is the autoregressive coefficient in the *AR*(*p*) model, and {*x*_*t*_} is the time series. The advantage of using this AR method is that it can find the occurrences of randomness in data. It can also predict any recurring patterns in the data. In this paper, the least-square estimation method is used to solve the model parameter *a*_*i*_. For the time series {*x*_*t*_}, when *j* ≥ *p* + 1, the estimate of *ε*_*t*_ is

(2) $$\begin{array}{c} \varepsilon_{j}=x_{j}-\left(a_{1}x_{j-1}+a_{2}x_{j-2}+\cdots +a_{p}x_{j-p}\right). \end{array}$$

This results in the following formula:

(3) $$\begin{array}{c} \sum_{j=p+1}^{N}{\left[x_{j}-\left(a_{1}x_{j-1}+a_{2}x_{j-2}+\cdots +a_{p}x_{j-p}\right)\right]}^{2}. \end{array}$$

The smallest *a*_1_, *a*_2_,…, *a*_*p*_ are the estimates of the autoregressive parameters *a*_1_*, a*_2_,…, *a*_*p*_ in the *AR*(*p*) model. In order to facilitate analysis, remember that

(4) $$\begin{array}{c} Y=\left[\begin{array}{c} x_{p+1}\\ x_{p+2}\\ M\\ X_{N} \end{array}\right],\\ X=\left[\begin{array}{cccc} x_{p} & x_{p-1} & \Lambda & x\\ x_{p+1} & x_{p} & \Lambda & x_{2}\\ M & M & O & M\\ x_{N-1} & x_{N-2} & \Lambda & x_{N-p} \end{array}\right],\\ a=\left[\begin{array}{c} a_{0}\\ a_{1}\\ M_{0}\\ a_{p} \end{array}\right],\\ \varepsilon =\left[\begin{array}{c} \varepsilon_{p+1}\\ \varepsilon_{p+2}\\ M\\ \varepsilon_{N} \end{array}\right]. \end{array}$$

We can get

(5) $$\begin{array}{c} Y=Xa+\varepsilon ,\\ S\left(a\right)={\left(Y-Xa\right)}^{T}\left(Y-Xa\right)=Y^{T}Y-2Y^{T}Xa+a^{T}X^{T}a. \end{array}$$

Taking the derivative of parameter *a* and setting it to zero, we get

(6) $$\begin{array}{c} \frac{\partial S\left(a\right)}{\partial a}=-2Y^{T}X+2a^{T}X^{T}X=0. \end{array}$$

Therefore, the least-square estimate of parameter *a* is

(7) $$\begin{array}{c} a={\left(X^{T}X\right)}^{-2}X^{T}Y. \end{array}$$

The least-square estimate of residual variance is

(8) $$\begin{array}{c} \sigma^{2}=\frac{1}{N=P}{\left(Y-Xa\right)}^{T}\left(Y-Xa\right). \end{array}$$

where *σ* is the extracted feature.

RETRACTED

#### 3.2.2. PCA-Based Abnormal Indicators

Principal Component Analysis is a feature extraction method. PCA avoids redundant features and provides unique features with minimum loss of original information. The abnormal index based on PCA is shown in the following equation:

(9) $$\begin{array}{c} \text{DI}=C*\underset{i\in n}{\max}\sqrt{\sum_{j=1}^{m}{\left[{\left(Z-Z*W*W^{T}\right)}^{2}\right]}_{i,j}}, \end{array}$$

where *Z* is the *n* × *m* input matrix, *n* is the number of training samples, *m* is the feature of the dimension of each instance, and *c* is the threshold coefficient.

### 3.3. Adolescent Health Data Mining Algorithm Based on Hadoop/Spark

Hadoop is an open-source big data platform that can run on low-cost hardware devices to provide applications with a distributed storage and computing environment across computer clusters to efficiently store and quickly compute large-scale data sets efficiently. With the storage layer (distributed file system, HDFS) and computing layer (MapReduce) as the core, Hadoop has become a widely used big data analysis platform due to its advantages of economy, reliability, scalability, and efficiency. Hadoop is the top level of Apache projects; after continuous development, it has produced many subprojects, which together constitute a fully functional Hadoop ecosystem, as shown in Figure 1.

1. HDFS architecture: Figure 2 shows the architecture diagram of HDFS. The NameNode is the master server (Master), which is mainly responsible for the management and operation of the namespace of the file system and at the same time controls the access of the client to the files. The DataNode is the slave node (Slave) responsible for storing and managing the data to be processed. The data operation of HDFS (Figure 2) is “write once, read many times.” Files in HDFS are usually divided into multiple data blocks with a size of 64 MB, and each data block is distributed to a different DataNode for storage. When a client wants to access a file, the client needs to obtain the DataNode memory map of each data block from the NameNode and then get the data block on the corresponding DataNode and finally obtain a complete data file.
2. Parallel computing framework MapReduce: the architecture of MapReduce is shown in Figure 3. The MapReduce cluster generally includes a Master and multiple SlaveMasters, and the Slave runs JobTracker service and TaskTracker service, respectively.
3. Spark architecture: Figure 4 shows the execution architecture of the Spark cluster. Apache Spark is a high-level and general-purpose cluster computing platform designed to be fast and fault-tolerant. It is an open-source big data processing and memory-efficient computation framework where the data is maintained and processed in shared physical memory. Spark is an efficient computational framework for iterative machine learning algorithms and supports multiple programming languages such as Python, Java, *R*, and Scala. The Spark architecture is comprised of a driver program, cluster manager Spark Context, and worker node. There is one primary/central coordinator in this architecture, and there are many distributed worker nodes. The primary/main coordinator is known as Spark Driver.

RETRACTED

Communication with all the workers is Spark Driver's responsibility. One or more executors are running on every worker node. Executors' job is to process the task. Executors have to register themselves with the Driver, and the Driver has all the information about Executors. A spark application is the working combination of Driver and Workers.

## 4. Experiments

This section gives detailed discussion on the experimental setup cluster construction and implementation of the proposed algorithm.

### 4.1. Experimental Environment

This article uses virtual machines and Docker virtualization technology to build a big data platform due to the limited experimental conditions. The virtual machine provides a Linux environment, and Docker serves as the running container of the cluster nodes. The hardware environment, software environment, and cluster node configuration of the cluster are shown in Table 3 and 4.

### 4.2. Docker-Based Hadoop/Spark Cluster Construction

The main steps of using Docker to deploy a Hadoop/Spark cluster are shown in Figure 5. The following focuses on the process of building a Hadoop cluster and a Spark cluster.

The first step is to install the Docker and pull the Centos image. In the next level, SSH, Hadoop, and Spark were established. In the third level, the Master and two Slaves were created, and finally the cluster is started.

### 4.3. Implementation of the Proposed Algorithm on Hadoop/Spark Platform

This paper uses the Apriori algorithm to give its distributed implementation on the Hadoop/Spark big data platform. Run the Apriori algorithm on a single machine and cluster with different nodes and test the algorithm's time to run. The result is shown in Figure 6. It can be seen from the figure that the Apriori algorithm takes 1192 s to run on a standard single machine. The running time on the big data platform has been dramatically shortened. As the cluster size increases, the running time gradually decreases, indicating that the distributed computing big data platform has good computing performance for data mining algorithms and can effectively improve the algorithm's computational efficiency.

## 5. Conclusion

This paper proposes using commonly used data mining algorithms and Hadoop/Spark big data processing platform to study and implement Hadoop/Spark-based structural health monitoring data mining algorithms. A comprehensive analysis of young students' physical fitness is provided through the mining of historical monitoring data and real-time monitoring data. Comparing the algorithm's running time on different platforms shows that the big data platform has good computing performance for the data mining algorithm. This research aims to establish a complete physical health data management system and effectively save, process, and analyze adolescents' physical test data through the system. After the analysis, on the one hand, it can provide students and schools with intuitive analysis results, and, on the other hand, it can be accurate. Reflect the specific problems of students in physical health to formulate specific measures to promote young people's physical fitness.

RETRACTED

## Figures and Tables

**Figure 1:** Hadoop ecosystem.

**Figure 2:** HDFS architecture.

**Figure 3:** MapReduce architecture.

**Figure 4:** Spark architecture.

**Figure 5:** Docker-based Hadoop/Spark cluster deployment flowchart.

**Figure 6:** Algorithm's running time on different platforms.

**Table 1:** Distribution of self-assessment status of adolescents' health.

Variable	Frequency	Percentage
Very good	332	38.5
Good	401	46.5
General	108	12.5
Have a chronic disease	21	2.5
Have a serious illness	1	0.1

**Table 2:** Analysis of the physical health of young people.

Variable	Mean	Std	Min	Max
Achieve 7–8 hours of healthy sleep per day	3.16	1.32	1	5
Achieve 0.5–1 hour of moderate-intensity aerobic exercise per day	3.09	1.22	5	5
No partial eclipse, eat three meals a day on time and according to the amount	3.71	1.21	5	5

Std = standard deviation, Min = minimum, Max = maximum.

**Table 3:** Experimental hardware platform and software simulation environment.

Hardware	Specification
CPU	Intel(R) Core(TM) i5-4200M CPU @ 2.50 GHz
RAM	8.00 GB
Operating system	Centos 8.0
Development environment	Hadoop 2.7
Spark	Spark 2.0

**Table 4:** Cluster node configuration.

Host	IP	Node type
Master	172.16.0.1	NameNode/Master
Slave 01	172.16.0.2	DataNode/worker
Slave 02	172.16.0.3	DataNode/worker

## Data Availability

The data used to support the findings of this study are included within the article.
